# Neuroprotective Effect of Acupuncture against Single Prolonged Stress-Induced Memory Impairments and Inflammation in Rat Brain via Modulation of Brain-Derived Neurotrophic Factor Expression

**DOI:** 10.1155/2022/4430484

**Published:** 2022-02-23

**Authors:** Bombi Lee

**Affiliations:** Acupuncture and Meridian Science Research Center, College of Korean Medicine, Kyung Hee University, 26, Kyungheedae-ro, Dongdaemun-gu, Seoul 02447, Republic of Korea

## Abstract

Posttraumatic stress disorder (PTSD) is a serious mental disorder that can appear after exposure to extreme stress. Acupuncture is an alternative therapy that is widely used to treat various neurodegenerative diseases, as well as cognitive and memory impairments. The aim of this study was to examine whether acupuncture stimulation at a specific acupoint (Shenmen or heart meridian, HT7) could improve memory defects caused by single prolonged stress (SPS) in rats. After exposure to SPS, acupuncture on the HT7 acupoint in male rats was performed, once daily for 21 days. We confirmed that this treatment improved fear memory, cognitive function, and spatial memory by modulating the neuroinflammation and expression of brain-derived neurotrophic factor (BDNF) mRNA in the brain. It also significantly inhibited the activation of proinflammatory cytokines, such as tumor necrosis factor-*α* and interleukin-1*β* and the enzyme cyclooxygenase-2 in the brain; it increased the expression of BDNF mRNA in the hippocampus. Our findings provide valuable information concerning the clinical usefulness of acupuncture in the treatment of PTSD.

## 1. Introduction

Posttraumatic stress disorder (PTSD) is a mental disorder in which fear memory and anxiety reactions appear after exposure to a previously experienced traumatic event (e.g., a car accident, disaster, abuse, or extreme stress) [1]. In particular, although the incidence rate of PTSD is increasing among the elderly, these symptoms of PTSD are often ignored or not recognized in the early stages of PTSD [2]. PTSD greatly reduces the quality of life of patients and causes psychiatric comorbidities [1, 2]. Unlike general stress, PTSD causes fear memory disorders to appear even in safe situations when the traumatic event has disappeared; it can cause serious pathological changes such as anxiety disorders, depression, flashbacks, and cognitive memory dysfunction [3].

PTSD is caused by excessive stress-related dysregulation of the hypothalamic-pituitary-adrenal (HPA) axis and neurophysiological imbalance in the fear circuit region of the brain [2, 4]. PTSD causes a breakdown of the immune system and excessive secretion of the stress hormone, corticosterone (CORT), by excessive release of proinflammatory cytokines by a neuroinflammatory response [5–8]. Therefore, in PTSD patients, proinflammatory cytokines (e.g., interleukin-1*β* (IL-1*β*) and tumor necrosis factor-*α* (TNF-*α*)) accumulate in large amounts in the fear circuit region of the brain, such as the medial prefrontal cortex (mPFC), hippocampus (Hipp), and amygdala (Amg) [9, 10]. This neuroinflammation causes fear memory and impairments of both cognitive function and spatial memory in PTSD [11, 12]. In particular, neuronal cell damage in the fear circuit region causes memory impairment through a decrease in brain-derived neurotrophic factor (BDNF), increases in proinflammatory cytokines, and changes in synaptic plasticity [13]. In an inflammatory response, cyclooxygenase-2 (COX-2) is a rate-limiting enzyme involved in prostaglandin E2 synthesis, which is regulated by proinflammatory cytokines [14]. COX-2 levels increase in both neurodegenerative and stress-related diseases; the administration of a COX-2 selective inhibitor inhibits the cell damage caused by oxidative stress in an animal model [15, 16]. Several studies have shown that COX-2 inhibitors inhibit apoptosis and increase inflammatory factors in a PTSD animal model [14].

Because a fundamental and effective treatment method is unavailable for the complex mechanism underlying PTSD, anti-depressants are used most frequently; these therapeutic agents have limitations related to their serious side effects and the potential for treatment refusal.

Acupuncture is widely used as an alternative medicine for the treatment of memory impairment, including mental disorders [17–19]. In addition, acupuncture is effective for balancing biochemical changes and maintaining or restoring homeostasis in the central nervous system [20]. Recently, acupuncture was found to be effective in improving the memory impairment caused by chronic stress and dysregulation of the HPA axis in rats [21]. Some studies have reported that low-frequency electrical stimulation of a specific acupoint (Shenmen or heart meridian, HT7) significantly improves anxiety-like behavior by reducing the stress-induced chronic production of CORT in rats; it also restores the expression of the neuropeptide Y and the gene c-Fos in the paraventricular nucleus of the hypothalamus [22]. Furthermore, acupuncture stimulation of HT7 reduces cerebral infarction damage by ischemic reperfusion and reduces the number of apoptotic neurons in the CA1 region of the Hipp of mice [23]. Many studies have supported the usefulness of acupuncture by showing that it can alleviate the stress-related behavioral and physiological components of memory function [2, 24, 25]. East Asian medical studies have shown that the HT7 acupoint is an important acupuncture point for alleviating neuroinflammation and memory impairment [25, 26]. Therefore, we hypothesized that acupuncture involving this acupoint may help improve cognitive impairment-related disorders caused by PTSD.

The present behavioral and neurochemical study analyzed the effects of acupuncture treatment on fear memory, cognitive function, and spatial memory impairment after single prolonged stress (SPS) in an animal model of PTSD. The effect of acupuncture was assessed by examining changes in the expression of proinflammatory cytokines in the mPFC, Hipp, and Amg, and COX-2 in neuroinflammatory responses and changes in BDNF expression in the Hipp.

## 2. Methods

### 2.1. Animals

We used male Sprague-Dawley rats (Samtaco Animal Co., Seoul, South Korea). Eight-week-old, 200∼250 g rats were allowed to adapt to the breeding conditions in the laboratory for one week; they were also accustomed to the experimenter via handling procedures. During the adaptation period, the rats lived in group breeding boxes of 3∼4 animals; the room was maintained at 23 ± 2°C with 40∼50% humidity. Sufficient food and sterile drinking water were provided; day and night lengths were artificially set to 12 h each. Considering the rats' nocturnal behavior, the night cycle was set to correspond to actual daytime throughout the experiment. Animal experiments were conducted in accordance with the Code of Ethics and guidelines for the management of laboratory animals by the Animal Care and Use Committee of Kyung Hee University (Seoul, South Korea), which also approved the experimental protocol (KHUASP(SE)-21-045).

### 2.2. Acupuncture Stimulation

Acupuncture stimulation was performed on both forefeet for 5 min every day after SPS, as previously described [25]. HT7 is located on the most medial axis of the transverse fold of the wrist of the forefoot. We selected the Zusanli (stomach median, ST36) acupoints and tail point stimulation as comparator acupoints and nonacupoints, respectively. ST36 is located approximately 8∼9 cm below the knee, in a hollow outside the tibia and inside the Achilles tendon. Tail point stimulation was performed at one-fifth of the length of the tail from its proximal end. We used sterile, disposable, stainless steel needles (0.18 mm × 20 mm, Suzhou Kangnian Medical Devices Co. Ltd., Suzhou, China). The needles were perpendicularly inserted to a depth of 2∼3 mm at HT7, ST36, or the tail point. During 2 sec of stimulation by insertion and withdrawal of the needle at the acupuncture point, acupuncture stimulation was delivered manually by twisting the needle at a frequency of twice per second. The insertion depth and anatomical position of each acupoint were determined from previous studies [25]. Rats were treated gently to ensure they experienced only minimal stress during the acupuncture stimulation process.

### 2.3. Single Prolonged Stress

In the SPS process, rats were subjected to restraint stress for 2 h and forced to swim for 20 min. Rats were allowed to rest for 15 min and then exposed to isoflurane (2∼3%) until they became unconscious. After SPS, the rats were left alone for 7 days for sensitization in the same manner as previously reported [27]. The detailed experimental schedule is shown in Figure 1.

### 2.4. Contextual Fear Conditioning and Extinction

For learned fear of sensory stimuli, we performed a conditioned fear test (CFT) using a fear conditioning box (30 cm × 30 cm × 30 cm). On day 1, rats were acclimatized for 1 min in the box, thereby initiating the adaptation trial. After 1 min, the rat was placed on the railing (5 cm × 15 cm) on the front outer wall of the box; a light (50 W) installed 45 cm above the railing was used to illuminate the rat. When the rat entered the box through a small sliding door (5 cm × 5 cm), the adaptation trial ended. The rat was returned to the railing and exposed to the light again. When the rat entered the fear conditioning box, a conditional stimulus (sound alarm: 30 sec, 85 dB) was applied. During the last 2 sec of the conditional stimulus, a single electric foot shock (0.5 mA, 2 sec) was applied (as an unconditional stimulus, forming the learning trial). This learning trial was repeated 3 times, with a 2 min rest period after each session (i.e., the intertrial interval). On day 2, when the rats entered the fear conditioning box from the railing, no conditional stimuli or shocks were applied, forming the extinction training. This extinction training was repeated 6 times. To test the contextual response, when rats entered the fear conditioning box from the railing, after exposure to the conditional stimulus alone, we observed the rat's fear response for 5 min. The fear response was the duration of the freezing response with no movement other than breathing.

### 2.5. Object Recognition Task

We performed an object recognition task (ORT) as previously reported [28]. The experimental apparatus consisted of a black acrylic box (40 cm × 40 cm × 25 cm). Habituation was performed by exposing each rat to the experimental apparatus for 5 min in the absence of the object. After 24 h of habituation, each rat was placed in the same context box with two similar wooden toys (familiar objects, A1 and A2) and allowed to explore for 5 min (i.e., object training). After a maintenance interval of 24 h, each rat was placed back into the same context box. One of the objects was replaced with a new wooden toy (B), and the rat was allowed to search for 5 min. In the ORT, the exploratory behavior of each rat was recorded to evaluate its navigation time; the time spent exploring each object (familiar and novel) was recorded. Preference for familiar objects was expressed as the percentage of time spent searching for new objects, compared with the total time spent searching for two objects.

### 2.6. Morris Water Maze Test

We performed a Morris water maze (MWM) test. The apparatus for this was a plastic circle water tank (15 cm in diameter and 20 cm in height) which was installed in the center of one quadrant of the tank. The tank was filled with water to a depth of 22 cm. A video camera was installed on the ceiling above the tank to record rats' movements during learning. At 30 min before the start of the experiment, a rat was transferred to the maze laboratory and acclimatized to the experimental conditions. Learning was conducted 3 times daily. The rat swam freely in the tank; the trial ended when the rat found the escape platform. If the rat did not find it within 180 sec, the experimenter gently guided the rat to the escape platform and ended the trial. The learning performance measured in each learning trial was the escape latency (i.e., the time required until the rat found the escape platform); we defined the maximum escape latency as 180 sec for rats that did not find the escape platform without guidance. When a rat climbed onto the escape platform either spontaneously or under the guidance of the experimenter, it was allowed to stay there for 10 sec. When that interval elapsed, we placed the rat at the center point of another quadrant, beginning the next trial. In this manner, rats were placed in each quadrant, and three trials were completed for each day of learning (i.e., each learning session). These sessions were repeated for 5 days. After the 5th learning session, we performed a memory test on the 6th day. In this test, the escape platform was removed from the tank, and each rat swam for 60 sec; we measured the time the rat spent in the target zone where the escape platform had been located (an area with a diameter of 40 cm centered on the escape platform) and the number of times it passed through the zone. We regarded these measures as scores of memory.

### 2.7. Open Field Test

When a rat is exposed to a new environment, it exhibits exploratory behavior; we measured the amount of the rat's locomotor activity as an index of this behavior. The apparatus used for this open field test (OFT) was a black wooden box (60 cm × 60 cm × 30 cm) illuminated by an incandescent light bulb (60 W) mounted on the ceiling 2 m above. A camera was installed on the ceiling above the center of the open field; the rat's behaviors were recorded and analyzed using SMART software (version 2.5; PanLab Co., Barcelona, Spain). At 30 min before the start of the experiment, the rats were moved to the behavioral observation room and acclimatized to the experimental conditions; locomotor activity was then recorded for 5 min. When each rat completed a behavioral experiment, the open field apparatus was wiped clean to remove the odor left by the rat.

### 2.8. Enzyme-Linked Immunoassay Analysis of Inflammatory Mediator Levels

After the behavioral test had been completed, four rats from each group were randomly selected and used for enzyme-linked immunosorbent assay (ELISA) measurement. The brains of the rats were immediately removed, and the mPFC, Hipp, and Amg tissues were separated. Each tissue was placed in Tris-HCl buffer, homogenized, and centrifuged. Proinflammatory cytokines (TNF-*α* and IL-1*β*) and COX-2 protein measurements were performed using commercial kits from Abcam (Cambridge, MA, USA) and Cell Signaling (Danvers, MA, USA). We conducted the assays in accordance with the manufacturers' instructions and repeated the measurements 3 times for each sample.

### 2.9. Total RNA Isolation and Reverse Transcription Polymerase Chain Reaction Analysis

We measured the expression levels of BDNF and tropomyosin receptor kinase B (TrkB) mRNA by reverse transcription polymerase chain reaction (RT-PCR). We rapidly removed the rats' brains and stored them at −80°C until use. Total RNA was prepared from the homogenized Hipp using 1 mL of TRIzol reagent (Invitrogen Co., Carlsbad, CA, USA). Complementary DNA was synthesized from total RNA using reverse transcriptase (Takara Co., Shiga, Japan). For polymerase chain reaction (PCR) analysis, primers specific for each mRNA sequence were used with a previously reported reagent [29]. PCR amplification was performed at 56°C for 28 cycles for BDNF and 57°C for 30 cycles for TrkB using a thermal cycler (MJ Research, Watertown, MA, USA). The PCR products were separated on a 1.2% agarose gel and stained with ethidium bromide. The density of each band was quantified using an image analysis system (i-MaxTM, CoreBio System Co., Seoul, South Korea). The expression levels were compared by calculating the relative density of each target band to the relative density of glyceraldehyde 3-phosphate dehydrogenase (GAPDH).

### 2.10. Statistical Analysis

All data are shown as means ± standard errors. Differences between groups were analyzed with SPSS software (version 23.0; SPSS Inc., Chicago, IL, USA) using one-way analysis of variance (ANOVA) and Tukey's post hoc test. A *p* value <0.05 was considered statistically significant.

## 3. Results

### 3.1. Changes in Body Weight and Serum CORT Level after SPS

We observed the rats' body weight for 21 days after SPS; in saline-treated (SAL) normal rats, the body weight gradually increased over time (Figure 2(a)). However, the SPS group showed little change in body weight from the 2nd day to the 7th day (*t* = 4.659, *p* < 0.01). Although the change in body weight gradually increased after the day 7 sensitization period, we found that this increase was significantly less than in the normal group. The body weight of the SPS group was 13.7% less than the body weight of the SAL group on day 21. This showed that there was a physiological change in the body weight because of the SPS-induced traumatic stress. However, rats treated with HT7 acupoint showed no significant difference in reduction in body weight gain compared with the SPS group.

We measured the serum CORT levels of rats after SPS (Figure 2(b)). The SPS group showed a significant increase, compared with the SAL group (*p* < 0.01). The HT7 acupoint group exhibited significant inhibition of SPS-induced increases in serum CORT levels (*p* < 0.05). The increased levels of CORT, a stress hormone, indicated that SPS elicited stress-induced dysregulation of the HPA axis in rats; this was alleviated by HT7 acupoint treatment.

### 3.2. Effect of Acupuncture on Freezing Response after SPS

There was no difference in the freezing response between SAL and SPS groups during conditioning (learning trial; *t* = 0.458, *p*=672; Figure 3(a)). However, during extinction training, the freezing response was significantly increased in the SPS group, compared with the SAL group (*t* = 4.371, *p* < 0.05). During extinction recall, the freezing response was also significantly increased in the SPS group, compared with the SAL group (*p* < 0.01; Figure 3(b)). However, the HT7 acupoint group showed a significant decrease in the freezing response to extinction recall, compared with the SPS group (*p* < 0.05). The ST6 acupoint and tail point stimulation groups did not significantly differ in their freezing responses to extinction recall (*p*=0.970 and *p*=0.999, respectively). Therefore, SPS induced a conditional fear response, and HT7 acupoint treatment improved the extinction of fear memory.

### 3.3. Effect of Acupuncture on Impairments of Cognitive and Spatial Memory after SPS

The sniffing time for familiar objects did not differ among the groups (*F*_4,34_ = 1.647; *p*=0.188; Figure 3(d)). However, the SPS group had a significantly lower sniffing time for new objects than did the SAL group (*p* < 0.001; Figure 3(e)). Furthermore, the HT7 acupoint group tended to show an increase in the sniffing time for a new object, compared with the SPS group, although this difference was not statistically significant (*p*=0.059). There were no significant differences in sniffing times for new objects between the ST6 acupoint and tail point stimulation groups, compared with the SPS group (*p*=0.709 and *p*=0.858, respectively).

Notably, the SPS group showed a significant decrease in the discrimination index, which is the ability to recognize new objects, compared with the SAL group (*p* < 0.01; Figure 3(f)). However, the HT7 acupoint group showed a significant increase in this index, compared with the SPS group (*p* < 0.05). There were no significant differences in the discrimination indexes of the ST6 acupoint and tail point stimulation groups, compared with the SPS group (*p*=0.344 and *p*=0.153, respectively). Therefore, SPS rats exhibited impaired cognitive memory ability, which was improved in the HT7 acupoint rats.

The ability to find the hidden platform was significantly worse in the SPS group than in the SAL group, with a higher escape latency during the 5-day training (acquisition) phase (*p* < 0.01 on days 3 and 4 and *p* < 0.001 on day 5; Figure 4(a)). However, the escape latency was significantly lower in the HT7 acupoint group than in the SPS group (*p* < 0.05 on day 4). Furthermore, neither the ST6 acupoint nor tail point stimulation affected the escape latency (*p*=0.362 and *p*=0.971 on day 4, respectively). In the escape latency on the 5th day of training, the HT7 acupoint group tended to exhibit improved learning ability, compared with the SPS group, although this difference was not statistically significant (*p*=0.126). However, during the 5-day training phase, the HT7 acupoint group exhibited a better ability to find the hidden platforms. There were no differences in mean swimming speed among the groups (*F*_4,30_ = 3.719; *p*=0.051; Figure 4(b)).

In the retention test to confirm spatial memory ability, we measured the percentage of time spent in the target zone with the escape platform removed, the percentage of distance travelled in the target zone, the number of entries to the target zone, and the time to initially enter the target zone (Figures 4(c)∼4(f)). The SPS group had significantly reduced percentages of time spent and distance travelled in the target zone, compared with the SAL group (*p* < 0.01, for both). However, the HT7 acupoint group showed significant increases in these measurements, compared with the SPS group (*p* < 0.05, for both). Furthermore, there were no significant differences in these measurements between the ST6 acupoint and tail point stimulation groups, compared with the SPS group (*p*=0.699, *p*=0.999, *p*=0.530, and *p*=0.097, respectively). Therefore, the SPS rats exhibited an impaired spatial memory ability, which was improved in the HT7 acupoint rats.

There were no differences in locomotor activity among the groups (*F*_4,34_ = 1.043; *p*=0.402; Figure 3(c)).

### 3.4. Effect of Acupuncture on Proinflammatory Cytokines in the mPFC, Hipp, and Amg after SPS

The SPS group had significantly increased levels of proinflammatory cytokines (TNF-*α* and IL-1*β*) in the mPFC and Hipp, compared with the SAL group (*p* < 0.05 and *p* < 0.001, respectively; Figures 5(a)∼5(f)). However, the HT7 acupoint group had significantly lower levels of TNF-*α* in the Hipp (*p* < 0.05; Figures 5(a) and 5(b)) and IL-1*β* in both mPFC and Hipp (*p* < 0.05; Figures 5(d) and 5(e)), compared with the SPS group. The SPS group tended to exhibit higher levels of TNF-*α* and IL-1*β* in the Amg, although these differences were not statistically significant (*p*=0.766 and *p*=0.091, respectively). Furthermore, the ST6 acupoint and tail point stimulation did not affect the proinflammatory cytokine levels in the mPFC, Hipp, or Amg, compared with the SPS group.

### 3.5. Effect of Acupuncture on COX-2 Level in the Hipp after SPS

The SPS group had a significantly higher level of COX-2 in the Hipp, compared with the SAL group (*p* < 0.05; Figure 5(g)); however, the HT7 acupoint group had a significantly lower level of COX-2 (*p* < 0.05). The ST36 acupoint and tail point stimulation did not affect the level of COX-2 in the Hipp (*p*=0.767 and *p*=0.435, respectively).

### 3.6. Effect of Acupuncture on the Expression Levels of BDNF and TrkB mRNAs in the Hipp after SPS

The SPS group had a significantly lower expression level of BDNF mRNA in the Hipp, compared with the SAL group (*p* < 0.05; Figure 6(a)); the HT7 acupoint group showed a significantly higher expression level of BDNF mRNA (*p* < 0.05). This expression level did not significantly differ in the ST6 acupoint and the tail point stimulation groups, compared with the SPS group (*p*=0.398 and *p*=0.164, respectively). The SPS group tended to exhibit lower expression of TrkB mRNA in the Hipp, compared with the SAL group, although this result was not statistically significant (*p*=0.053; Figure 6(b)); the HT7 acupoint group also tended to exhibit an increase that was not statistically significant (*p*=0.233).

## 4. Discussion

Our results confirmed the effects of acupuncture treatment on the fear memory, cognitive function, and spatial memory impairments caused by neuroinflammation in an animal model of PTSD. Acupuncture focused on the HT7 acupoint restored the ability to extinguish the fear memory caused by traumatic stress in SPS-exposed rats; it also improved spatial learning and reduced memory impairment. Furthermore, it showed an anti-inflammatory effect in the exaggerated inflammatory condition after immune system disruption, regulating the increase in COX-2 and decrease in BDNF. Therefore, the present study confirmed that acupuncture focused on the HT7 acupoint could be useful for the treatment of fear memory, memory impairment, and neuroinflammation in PTSD.

In our study, SPS-exposed rats showed weight loss and increased serum CORT levels. In animal models of PTSD, high concentrations of CORT and weight loss caused by dysregulation of the HPA axis are physiological features common with PTSD patients [30]. A high concentration of CORT caused by a response to traumatic stress causes increased levels of proinflammatory cytokines, failure to extinguish fear memories, and behavioral changes related to memory dysfunction [12]. Therefore, the reduction of serum CORT from acupuncture focused on the HT7 acupoint suggests the possibility of recovery from the behavioral response and neuroinflammation caused by memory impairment.

Neuronal cell damage to the mPFC, Hipp, and Amg (i.e., the fear circuit region of the brain) caused by PTSD impairs the acquisition of fear-extinction learning [31]. Our results showed that in the CFT, SPS-exposed rats had significantly increased freezing behavior after traumatic contextual fear and fear response during the extinction recall. However, acupuncture focused on the HT7 acupoint led to a decrease in freezing behavior after the weakening of fear in short-term extinction recall. Therefore, this acupuncture caused improvement in behavior after fear memory because of an improvement in the ability to extinguish fear.

We used the MWM test to assess spatial working memory and learning in an animal model of PTSD showed that such rats had impaired abilities in terms of spatial learning, well as consolidating and retrieving reference memories [32]. SPS-exposed rats exhibited a longer time to reach the escape platform, as well as decreased time and distance in the target quadrant, compared with normal rats. In addition, SPS rats spent more time in the quadrant opposite to the target zone. Our results in the MWM test were consistent with findings in previous studies, indicating that SPS-exposed rats develop learning and memory deficits during the acquisition phase. However, acupuncture focused on the HT7 acupoint restored the ability to maintain spatial learning and memory formation; it shortened the escape latencies while increasing the time and distance in the target quadrant.

Cognitive memory impairment caused by PTSD may reduce the preference for novelty [29]. SPS-exposed rats showed decreases in sniffing time and discrimination index with respect to novel objects. This is consistent with the hypersensitivity and increased neuro-fear circuit activation in PTSD patients who are exposed to new and potentially threatening stimuli [12, 33]. However, acupuncture focused on the HT7 acupoint led to improvements in cognitive memory impairment, such that these indicators were restored. Therefore, such acupuncture can elicit behavioral flexibility during the traumatic stress-induced fear response by improving the cognitive memory impairments that affect familiar and new stimuli.

To determine whether the SPS-induced cognitive memory and spatial memory impairments in rats were clearly linked to a decrease in movement caused by motor dysfunction, we assessed locomotor activity in all rats in the OFT; the results showed no significant differences among groups. These mean swimming speeds of rats in the MWM test were also consistent across groups. Therefore, the findings indicate that the additional time needed for rats to reach the platform and explore new objects was related to behavioral changes caused by memory impairment.

Traumatic stress stimulates the immune system to release proinflammatory factors, and it is known that excessive expression of inflammatory cytokines leads to neuronal cell damage in the fear circuit region of the brain, as well as pathological changes associated with PTSD [34]. Our results show that increases in TNF-*α* and IL-6 levels because of SPS exposure may have important roles in PTSD pathogenesis. The levels of the traumatic stress-induced proinflammatory cytokines TNF-*α* and IL-1*β* were significantly higher in the mPFC and Hipp. However, acupuncture focused on the HT7 acupoint significantly reduced the SPS-induced expression of IL-1*β* in the mPFC and Hipp; this approach significantly reduced the TNF-*α* level only in the Hipp. Notably, there were no differences in cytokine levels in the Amg after SPS. The Amg constitutes the fear circuit region of the brain, in combination with the mPFC and Hipp; however, the profile of cytokines affected by SPS appears inconsistent among brain regions. Furthermore, although acupuncture focused on the HT7 acupoint extinguished fear memory and improved spatial memory impairment because of reductions in the cytokine levels, these changes differed depending on the brain region. Our results have demonstrated that acupuncture focused on the HT7 acupoint may be more effective for relieving neuroinflammation in the mPFC and Hipp than in the Amg. These results are more dependent on the mPFC and Hipp than the Amg concerning the recovery of learning and memory; we presume that neuroinflammatory changes in the mPFC and Hipp contribute to pathological recovery after fear memory abnormalities. Moreover, the mPFC and Hipp, which respond effectively to acupuncture focused on the HT7 acupoint, are brain regions related to learning and memory. Therefore, based on our findings in this study, we suspect that acupuncture focused on the HT7 acupoint can sufficiently restore memory function through anti-inflammatory effects in the mPFC and Hipp, without regulation of the Amg.

In addition, SPS-exposed rats showed an increased level of COX-2 in the Hipp. However, this PTSD-induced increase was significantly improved by acupuncture focused on the HT7 acupoint. These results are consistent with previous findings that the inhibition of COX-2 reduced various types of stress-related memory dysfunction in rats [14]. The level of COX-2 protein is closely related to neuroinflammation *in vivo*; increases in TNF-*α* and IL-6 expression can be inhibited by a decrease in the COX-2 level [35]. This suggests that a feedback loop may exist between COX-2 and neuroinflammation [36, 37]. Our findings indicate that increased COX-2 expression is involved in the pathogenesis of PTSD; COX-2 may constitute a target for PTSD treatment. Moreover, acupuncture focused on the HT7 acupoint can improve memory impairment by inhibiting COX-2 production and inhibiting neuroinflammation in the Hipp of SPS-exposed rats.

BDNF, acting via TrkB, has an important role in neuroinflammation and memory function [38]. In animal models of PTSD, the response to traumatic stress is accelerated by increased inflammatory cytokine expression, which is caused by BDNF reduction. SPS-exposed rats were previously found to exhibit decreased BDNF expression and increased proinflammatory cytokine expression in the Hipp [39]. In our study, the reduction of BDNF after SPS exposure led to increases in proinflammatory cytokines (e.g., TNF-a and IL-1*β*) in the mPFC and Hipp, the fear circuit region of the brain. However, the regulation of BDNF in the Hipp by acupuncture focused on the HT7 acupoint was sufficient to alleviate the fear-induced abnormal behavior and restore both cognitive function and spatial memory; these changes were related to the anti-inflammatory effect of this acupuncture approach.

In our study, we showed that fear extinction failure and impairments of both cognitive function and spatial memory were associated with neuroinflammation and reduced BDNF expression. However, we found that changes in neuroinflammation and BDNF expression caused by acupuncture focused on the HT7 acupoint were involved in the improvement of fear extinction. These effects were demonstrated by the reduction of fear-related freezing behavior and the restoration of abilities to learn and consolidate memory because neuronal cells were protected in the fear circuit region of the brain.

## 5. Conclusion

Our results suggest that acupuncture is a potential treatment for PTSD-induced fear memory and impairments of both cognitive function and spatial memory in an SPS model. They also show that acupuncture inhibits neuroinflammation by reversing changes in the levels of proinflammatory cytokines and by regulating the levels of COX-2 and BDNF in the Hipp. The results of this study will be helpful to provide valuable information concerning the clinical potential of acupuncture in the treatment of PTSD; they will also be useful for investigating the role of neuroinflammation caused by PTSD.

## Figures and Tables

**Figure 1:** Experimental protocols for single prolonged stress (SPS)-induced memory impaired behavior and acupuncture treatment in rats. Different groups of rats (*n* = 6∼7/group) were used for each experimental condition. ORT: object recognition task and OFT: open field test.

**Figure 2:** Results of the body weight (A) and serum corticosterone (CORT) levels (B) of rats exposed to SPS for 21 days. Body weights are significantly lower in SPS-exposed rats than in saline-treated (SAL) normal rats (significant main effect of SPS exposure versus saline-treated rats). Data are presented as means ± standard errors of the mean.  ^*∗∗*^*p* < 0.01;  ^*∗∗∗*^*p* < 0.001 versus SAL group; and ^#^*p* < 0.05 versus SPS group.

**Figure 3:** Effects of acupuncture on freezing behavior in response to conditioning (C1∼C3), extinction (E1∼E6), and short-term recall (R1) (a) and the percentage of time spent frozen during short-term recall (b) in the contextual fear conditioning; on the travel distance of locomotor activity in the open-field test (c); and on exploration time to two familiar objects (d) and familiar and new objects (e), and the ability to discriminate between familiar and new objects (f) in the novel object recognition test.  ^*∗*^*p* < 0.05,  ^*∗∗*^*p* < 0.01,  ^*∗∗∗*^*p* < 0.001 versus SAL group, and ^#^*p* < 0.05 versus SPS group.

**Figure 4:** Effect of acupuncture on time to escape (latency) from the water onto a submerged platform during the acquisition trials (a), swimming speed (b), percentage of time spent in the target quadrant (c), percentage of distance travelled in the target quadrant (d), latency to reach the target zone (e), and number of entries to the target zone (f) in the Morris water maze.  ^*∗∗*^*p* < 0.01,  ^*∗∗∗*^*p* < 0.001 versus SAL group, and ^#^*p* < 0.05 versus SPS group.

**Figure 5:** Effects of acupuncture on tumor necrosis factor-*α* (TNF-*α*) expression in the medial prefrontal cortex (mPFC; (a)), hippocampus (Hipp; (b)), and amygdala (Amg; (c)); on interleukin-1*β* (IL-1*β*) expression in the mPFC (d), Hipp (e), and Amg (f); and on cyclooxygenase-2 (COX-2; (g)) expression in the Hipp of rats exposed to SPS according to enzyme-like immunosorbent assay analysis.  ^*∗*^*p* < 0.05,  ^*∗∗∗*^*p* < 0.001 versus. SAL group, and ^#^*p* < 0.05 versus SPS group.

**Figure 6:** Effect of acupuncture on the expression levels of brain-derived neurotrophic factor (BDNF; (a)) and tropomyosin receptor kinase B (TrkB; (b)) mRNAs in rats with SPS-induced memory impairment. The relative intensities of polymerase chain reaction amplification product bands on agarose gels are shown. The expression levels of BDNF and TrkB mRNAs were normalized to the expression level of glyceraldehyde 3-phosphate dehydrogenase mRNA as an internal control.  ^*∗*^*p* < 0.05 versus SAL group and ^#^*p* < 0.05 versus SPS group.

## Data Availability

All data supporting the conclusions of this article are included within the article. The data sets used/or analyzed during the current study are available from the corresponding author on reasonable request.
